# Efficacy and Safety of Transurethral Columnar Balloon Dilation of the Prostate for the Treatment of Benign Prostatic Hyperplasia: A Multicenter Trial

**DOI:** 10.1155/2022/7881247

**Published:** 2022-06-09

**Authors:** Guoyun Zhou, Jinkui He, Guangyi Huang, Ligang Ren, Wensong Zhuge, Wei Wang

**Affiliations:** ^1^Department of Urology Surgery, Zhejiang Lanxi Hospital of Traditional Chinese Medicine, Lanxi, Zhejiang 321102, China; ^2^Department of Urology Surgery, Zhejiang Yiwu Hospital of Traditional Chinese Medicine, Yiwu, Zhejiang 322015, China; ^3^Department of Urology Surgery, The Fourth Affiliated Hospital of Medical College of Zhejiang University, Hangzhou, Zhejiang 310030, China; ^4^Department of Urology Surgery, Zhejiang Provincial Tongde Hospital, Hangzhou, Zhejiang 310012, China

## Abstract

**Objective:**

To observe the efficacy and safety of transurethral columnar balloon dilation of the prostate (TUCBDP) for benign prostatic hyperplasia (BPH) in a multicenter trial.

**Method:**

This multicenter study included 2050 patients with BPH who underwent TUCBDP from 11 cities of Zhejiang Province, from September 2015 to June 2021. Clinical assessment included recording and measurement of preoperative and postoperative data including prostate volume, serum prostate-specific antigen (PSA) levels, IPSS score, quality of life (QoL), maximum urinary flow rate (Qmax), postvoid residual urine (PVR), International Index of Erectile Function (IIEF-5), and Male Sexual Health Questionnaire-Ejaculatory Dysfunction Short Form (MSHQ-EjD-SF). Additionally, the correlation of the indicators was analyzed using linear regression and early postoperative complications were also recorded.

**Results:**

One month after surgery, the patients' IPSS score, QoL, and PVR were significantly decreased, while the Qmax, IIEF-5, and MSHQ-EjD-SF scores were increased considerably, compared with preoperative data. After surgery, the patient's IPSS score, QoL, and Qmax were improved year by year, while PVR gradually decreased. Three months after TUCBDP, IIEF-5 and MSHQ-EjD-SF levels reached the climax. Linear regression analysis showed that the serum PSA level was significantly positively correlated with Qmax at 3 months after TUCBDP, while at 6 months after surgery, it was negatively related to IPSS and QoL. Early postoperative complications appeared in 384 cases during follow-up.

**Conclusion:**

Collectively, TUCBDP may effectively improve the urinary and sexual function of BPH patients, with fewer postoperative complications, and its efficacy is not limited by age and prostate volume. It can be considered a better treatment option for BPH.

## 1. Introduction

Benign prostatic hyperplasia (BPH) is one of the most common benign urogenital lesions in most middle-aged and elderly men. Its incidence and detection rates have increased year by year [1, 2]. Studies have found that the incidence of BPH is associated with age, which is more than 30% of people over 50 years old, about 50% in people over 60 years of age, and more than 80% in people aged over 80 years [3]. The early symptoms of BPH are characterized by increased nocturia, followed by a gradual onset of symptoms such as frequent urination, urgent micturition, dysuria, and even urinary retention [4]. This disease seriously affects the quality of life of patients and can even trigger a mental illness. Currently, there are active and minimally invasive procedures for the treatment of BPH, but the advantages of minimally invasive procedures with low rates of adverse events and rapid recovery have become the current preference. The following centralized options are usually available clinically: microwave transurethral thermotherapy (Tumt), transurethral prostate ablation (Tuna), prostate stenting, and prostatic urethral lift (PUL), but they also have significant disadvantages. For example, Tumt is not suitable for elderly patients with a high risk of anesthesia/surgery, and transurethral prostate ablation is not suitable for isolated obstruction of the prostate >75 ml [5–7]. In recent years, transurethral resection of the prostate has been recognized as the first-line surgical approach for BPH. Still, this procedure is reported to have disadvantages of a high incidence of complications such as postoperative bleeding, urethral stricture, resection syndrome, bladder neck injury, and retrograde ejaculation [8–10]. Therefore, active surgery and minimally invasive surgical treatment have become the main ways to relieve urinary tract symptoms and reduce related complications effectively.

In recent years, transurethral columnar balloon dilation of the prostate (TUCBDP), a new surgical procedure independently researched and developed in China, has gradually emerged as an option for BPH and has provided new concepts and ideas different from the traditional surgery [11]. This technology is simple and easy to learn, which can not only completely preserve the prostate but also has the characteristics of minor trauma, short operation time, less intraoperative blood loss, rapid postoperative recovery, especially its advantage of preserving the patients' sexual function, and achieved good short-term results in a study of 265 patients and confirmed a low complication rate (20%) for patients of advanced age who require preservation of sexual function, but the incidence of postoperative transient urinary incontinence (10.56%) appears to be high [12]. However, due to the lack of clinical applications, there is still considerable controversy about the indications and efficacy of TUCBDP [13]. Therefore, we analyzed the preoperative and postoperative follow-up data of 2050 patients with BPH who underwent TUCBDP. This multicenter study was conducted in 11 cities of the Zhejiang Province, and the selected patients were those treated between September 2015 and June 2021. Linear regression analysis was used to evaluate the clinical efficacy of TUCBDP and its surgical complications and postoperative sexual function were recorded and summarized to provide theoretical support for the clinical application and promotion of TUCBDP.

## 2. Material and Methods

### 2.1. General Information

The clinical data of patients with BPH who underwent TUCBDP in a multicenter study within 11 cities in Zhejiang Province, China, from September 2015 to June 2021 were collected. All enrolled patients had a definite diagnosis with an International Prostate Symptom Score (IPSS) ≥8. The age of the patients ranged from 55 to 93 years old with a medical history of 1-20 years. The main observation indicators at admission included prostate volume (PV), serum prostate-specific antigen (PSA) level, IPSS score, quality of life (QoL) score, maximum urinary flow rate (Qmax), postvoid residual urine volume (PVR), International Index of Erectile Function (IIEF-5), and Male Sexual Health Questionnaire-Ejaculatory Dysfunction Short Form (MSHQ-EjD-SF).

The patients included in this study had been screened strictly in accordance with the inclusion and exclusion criteria. To be specific, inclusion criteria were [14, 15] (1) patients with BPH who had failed to respond to conservative treatment, drugs, and other treatments and required surgery; (2) with complete inpatient diagnosis and treatment data; (3) PV of 30-150 mL; (4) IPSS score of 28 points, Qmax of 15 mL/s; (5) with other diseases such as bladder stones and urinary retention; (6) PSA<4 ng/mL, and prostate cancer was excluded before surgery in patients with an abnormal PSA level. Exclusion criteria included (1) patients diagnosed with prostate cancer, bladder cancer, and urethral cancer; (2) patients with severe heart, lung, brain diseases, patients with abnormal coagulation function or other severe systemic diseases, and patients unable to tolerate anesthesia and surgery; (3) patients with hyperplasia of the middle lobe, the distance from the tip of the prostate's protrusion into the bladder over 2 cm revealed by B-ultrasound examination, giant bladder diverticula; (4) patients with urethral stones or urinary tract infections.

Patient general information was recorded. Informed consent was signed by all patients, and this study was approved by the Committee of Zhejiang Lanxi Hospital of traditional Chinese Medicine.

### 2.2. Surgical Methods

Surgery was performed as described by Jia et al. [16]. Firstly, the transurethral catheter was selected based on the prostate size determined by B-ultrasound. Then, the patients were placed in the lithotomy position with low epidural anesthesia combined with spinal anesthesia. After that, the catheter was inserted into the bladder through the urethra. As the catheter was held in the left hand of a physician, the right index finger was used for digital examination of the rectum. After the fingertip touched a locating protrusion at the prostate apex, the catheter was pulled 1-1.5 cm outwards and fixed. The index finger and thumb were pinched in the rectum. After the thumb touched the locating protrusion in the perineum, 5-10 mL of normal saline was slowly injected into the balloon to maintain the pressure at 0.3 MPa. A water injection tube was then clamped to maintain the pressure for 5 minutes. The tube was periodically released 6 hours after surgery to reduce the water pressure gradually.

### 2.3. Observation Indicators

The prostate volume, serum PSA levels, IPSS scores, QoL, Qmax, PVR, IIEF-5, and MSHQ-EjD-SF were counted and analyzed before and after surgery.

### 2.4. Follow-Up

Follow-up was performed at 1, 3, 6, and 12 months postoperatively and annually thereafter until October 2021. During follow-up, IPSS score, QoL, Qmax, PVR, IIEF-5, and MSHQ-EjD-SF were recorded, and patients were asked if they were satisfied with their urinary function.

### 2.5. Postoperative Complications

The patients' occurrence of gross hematuria, hematospermia, dysuria, temporary urinary incontinence, urinary retention, urethral injury, and urinary tract infection were observed and recorded postoperatively. Whether the condition recurred was determined at the last follow-up.

### 2.6. Statistical Analysis

All data was analyzed using SPSS 24.0 statistical software. Measurement data were expressed as mean ± standard deviation (SD), and a paired *t*-test was used for comparison between two groups. Linear regression was also used to analyze the correlation of indicators in BPH patients. *P* < 0.05 was regarded as a statistically significant difference.

## 3. Results

### 3.1. Patient General Information

A total of 2050 patients were included, with an average age of (73.04 ± 10.78) years, a body mass index of 27.50 ± 2.21, PV of 51.23 ± 31.70 mL, a serum PSA level of 6.74 ng/mL, an IPSS score of 21.47 ± 3.46, QoL of 4.54 ± 1.09, Qmax of 8.91 ± 3.13 mL/s, PVR of 180.69 ± 44.33 mL, IIEF-5 of 20.96 ± 2.03, and MSHQ-EjD-SF of 10.47 ± 1.72 (Table 1).

### 3.2. Comparison of Prostatic Hyperplasia-Related Indicators in Patients before and after Surgery

The BPH-related indicators were detected before and after the surgery. Compared with the condition before treatment, the patients' IPSS score, QoL, and PVR at 1 month after surgery were significantly reduced and the Qmax, IIEF-5, and MSHQ-EjD-SF scores increased considerably. And over time, the IPSS score, QoL, and Qmax increased annually. At the last follow-up, the patient's IPSS score and Qmax were slightly lower than those at 12 months after surgery, while the QoL score was slightly higher than those at 12 months after surgery. PVR gradually decreased with follow-up time, with the level at the last follow-up slightly higher than that at 12 months after surgery. In addition, IIEF-5 and MSHQ-EjD-SF levels were at their highest at 3 months after surgery (Table 2).

### 3.3. Correlation Analysis of Prostatic Hyperplasia-Related Indicators in Patients

Linear regression analysis was used to analyze the correlation of prostate hyperplasia-related indicators. The results showed no significant correlations were found in patients' preoperative age, PV, postoperative IPSS scores, QoL, Qmax, and PVR throughout the follow-up. However, at 3 months after surgery, serum PSA level was significantly positively correlated with Qmax at 3 months after surgery and was negatively correlated with IPSS and QoL at 6 months after surgery (Figures 1(a)–1(l)).

### 3.4. Postoperative Complication in Patients

The occurrence of postoperative complications was statistically analyzed (Table 3). The results showed gross hematuria appeared in 12 BPH patients, hematospermia in 125 cases, dysuria in 36 patients, temporary urinary incontinence in 68 patients, urinary retention in 152 patients, urethral injury in 69 patients, and urinary tract infection in 19 cases. And hematospermia and urinary retention had the highest number of cases. The total cases of recurrence were 384, with an incidence rate of 18.7%.

## 4. Discussion

A pharmacological treatment can be administered for early stage of BPH, and common therapeutic drugs include *α*1 adrenergic receptor blockers [17], 5*α* reductase inhibitors [18], M receptor antagonists [19], and some herbal preparations [20]. Although drug therapy can relieve patients' clinical symptoms, slow disease development, and delay BPH-related complications, long-term use of drugs will lead to adverse reactions such as blood pressure fluctuations [21], loss of libido [18], constipation [22], and poor compliance with medical orders [23]. Surgical treatment can fundamentally relieve clinical symptoms by removing part of the hyperplastic glands, especially the transurethral resection of the prostate which effectively treats BPH. However, surgery still has limitations, such as inducing adverse reactions (prostate resection syndrome, bleeding, postoperative urinary incontinence, and retrograde ejaculation) [24–26]. Rapid development of science and technology has witnessed emergence of new surgical methods for BPH, such as plasmakinetic resection [27], laser surgery [28], and enucleation surgery [29]. But these operations have not been widely used due to the high requirements of patients' physical condition and expensive surgical equipment [30]. As a result, many elderly and high-risk BPH patients receive conservative treatment, such as the long-term wearing of the cystostomy tube, which has seriously reduced patients' quality of life and increased the incidence of infection and other related complications [30]. TUCBDP is the self-developed treatment method developed by the scientific research team led by Academician Guo Yinglu. It is a simple, safe, and effective new minimally invasive surgical method to treat BPH when this technology can effectively preserve normal organ function [31]. TUCBDP uses a columnar balloon to tear the surgical capsule of prostate and some prostate glands and widen the urethra of the prostate, thus improving urination symptoms. It has the advantages of short operation time, less bleeding, and preservation of the prostate with fewer complications, providing novel insight into BPH management [32]. However, there is currently a lack of long-term and large-scale clinical studies on patient conditions after TUCBDP, as most existing reports related to TUCBDP only have small samples within a short time period. In this study, by analyzing the efficacy of TUCBDP in 2050 BPH patients, we found that TUCBDP could effectively treat BPH with fewer postoperative complications, which is consistent with the results of the study by Xing et al. [33], However, it is inconsistent with the results reported by Wang et al. [12], which reported postoperative transient urinary incontinence as the most prevalent complication, whereas our findings suggest hematospermia and urinary postoperative morbidity as the most prevalent complication.

Urinary flow rate is the amount of urine excreted per unit time, resulting from the interaction between the detrusor contraction and urine outflow resistance. Of several indexes, Qmax acts as the most sensitive and significant parameter in measuring urinary flow rates. Compression of the enlarged prostate on the urethra may induce obstruction of the bladder outlet and increased urine outflow resistance, causing a decrease in Qmax and an increase in PVR [34]. Qmax, PVR, and IPSS scores in return are parameters reflecting and predicting the clinical progress of BPH. In this study, compared with the data before surgery, postoperative BPH patients had significantly decreased IPSS score, QoL, and PVR, significantly increased Qmax, and improvements in IIEF-5 and MSHQ-EjD-SF scores. At the last follow-up, patients had a high satisfaction rate with urinary function and sexual function. The above results suggest that TUCBDP can significantly improve prostate symptoms, quality of life, urinary tract obstruction symptoms, and urinary function with less impact on sexual function.

PSA is an androgen-regulated serine protease produced in prostate epithelial cells and prostate cancer. It is considered the most widely used serological diagnostic marker for prostate cancer and can be detected in male semen. As the most important protein in semen, PSA allows semen to become coagulated [35]. In this study, a significant positive correlation was found between serum PSA level and Qmax while PSA was negatively associated with IPSS and QoL. The above results suggest that serum PSA may be involved in regulating the malignant biological behavior of the prostate, but the specific mechanism needs to be confirmed by further research.

## 5. Conclusion

To sum up, TUCBDP can significantly improve the symptoms of lower urinary tract obstruction in patients with BPH with little impact on sexual function and fewer complications. In addition, not limited by age and PV, TUCBDP has good clinical efficacy and is a better choice for treating BPH. Serum PSA level may contribute to the malignant biological behavior of the prostate, but its specific mechanism needs to be further studied.

## Figures and Tables

**Figure 1:** Linear regression analysis. (a–d) Linear regression analyses of the correlations of age with IPSS (a), QoL score (b), Qmax (c), and PVR (d); (e–h) linear regression analyses of the correlations of prostate volume with IPSS score (e), QoL score (f), Qmax (g), and PVR (h); (i–l) linear regression analyses of the correlations of serum PSA level with IPSS score (i), QoL score (j), Qmax (k), and PVR (l).

**Table 1:** Patient general information.

Features	Mean ± SD	Median	Range
Age (year)	73.04 ± 10.78	74	10-42
Prostate volume (mL)	51.23 ± 31.70	43	8-381
Body mass index	27.50 ± 2.21	27.54	18.33-31.02
Serum PSA levels (ng/mL)	6.74 ± 3.97	6.7	0.46-42.26
IPSS scores	21.47 ± 3.46	22	16-32
QoL	4.54 ± 1.09	5	3-6
Qmax (mL/s)	8.91 ± 3.13	8.81	3.56-14.36
PVR (mL)	180.69 ± 44.33	179.27	105.12-255.88
IIEF-5	20.96 ± 2.03	21	13-25
MSHQ-EjD-SF	10.47 ± 1.72	10	8-13

Note: QoL: quality of life; Qmax: maximum urinary flow rate; PVR: Postvoid Residual Urine Volume; IIEF-5: International Index of Erectile Function; MSHQ-EjD-SF: Male Sexual Health Questionnaire-Ejaculatory Dysfunction Short Form.

**Table 2:** Comparison of benign prostatic hyperplasia related indicators in patients before and after surgery.

	IPSS	QoL	Qmax	PVR	IIEF-5	MSHQ-EjD-SF
Presurgery	21.47 (16-32)	4.54 (3-6)	8.91 (3.56-14.36)	180.69 (105.12-255.88)	20.96 (13-25)	10.47 (8-13)
1 month	18.94 (12-31)	3.99 (1-6)	11.20 (4.97-17.43)	158.37 (76.27-238.99)	21.46 (14-26)	10.50 (8-15)
3 months	20.92 (13-33)	4.08 (2-6)	13.58 (6.40-20.37)	135.99 (50.27-222.67)	21.96 (14-26)	11.46 (8-16)
6 months	22.54 (14-35)	4.89 (3-6)	15.81 (8.12-22.73)	113.55 (15.69-206.72)	21.67 (13-27)	11.09 (6-16)
12 months	25.96 (16-37)	4.62 (2-6)	18.11 (10.02-25.48)	91.32 (2.97-187.46)	21.42 (12-27)	10.93 (6-16)
Last follow-up	24.98 (16-37)	4.77 (1-6)	19.10 (11.35-26.68)	99.71 (10.82-194.99)	21.3 (12-28)	10.65 (5-17)
Changes from presurgery	+16.35	+5.51	+115.49	-44.82	+1.91	+1.72
*P*	≤0.001	≤0.001	≤0.001	≤0.001	≤0.001	≤0.001

Note: QoL: quality of life; Qmax: maximum urinary flow rate; PVR: Postvoid Residual Urine Volume; IIEF-5: International Index of Erectile Function; MSHQ-EjD-SF: Male Sexual Health Questionnaire-Ejaculatory Dysfunction Short Form.

**Table 3:** Statistics of postoperative complications.

Postoperative complications	*N*
Gross hematuria	12
Hematospermia	125
Dysuria	36
Temporary urinary incontinence	68
Urinary retention	152
Urethral injury	69
Urinary tract infection	19
Total cases of recurrence	384^∗^

^∗^The data is the total number of patients with recurrent symptoms (two or more conditions in a single patient).

## Data Availability

The data used to support the findings of this study are available from the corresponding author upon request.

## Abbreviations

BPH: Benign prostatic hyperplasia
TUCBDP: Transurethral columnar balloon dilation of the prostate
PSA: Prostate-specific antigen
IPSS: International Prostate Symptom Score
QoL: Quality of life
Qmax: Maximum urinary flow rate
PVR: Postvoid residual urine
IIEF-5: International Index of Erectile Function
MSHQ-EjD-SF: Sexual Health Questionnaire-Ejaculatory Dysfunction Short Form
Tumt: Microwave transurethral thermotherapy
Tuna: Transurethral prostate ablation
PUL: Prostatic urethral lift.
